# Transforming Growth Factor Beta Receptor 2 (TGFBR2) Promoter Region Polymorphisms May Be Involved in Mandibular Retrognathism

**DOI:** 10.1155/2022/1503052

**Published:** 2022-06-15

**Authors:** Margarita Kirschneck, Nermien Zbidat, Eva Paddenberg, Caio Luiz Bitencourt Reis, Isabela Ribeiro Madalena, Maria Angélica Hueb de Menezes-Oliveira, César Penazzo Lepri, Peter Proff, Christian Kirschneck, Erika Calvano Küchler

**Affiliations:** ^1^Department of Orthodontics, University of Regensburg, Regensburg, Germany; ^2^Department of Pediatric Dentistry, School of Dentistry of Ribeirão Preto, University of São Paulo, Ribeirão Preto, Brazil; ^3^Department of Dentistry, University of Joinville Region, Joinville, Brazil; ^4^School of Dentistry, Presidente Tancredo de Almeida Neves University Center, São João del Rei, Brazil; ^5^Department of Restorative Dentistry, School of Dentistry, Federal University of Juiz de Fora, Juiz de Fora, Brazil; ^6^Department Master's Program of Dentistry, School of Dentistry of Uberaba, Uberaba, Brazil

## Abstract

Skeletal malocclusions are common phenotypes in humans and have a strong influence on genetic factors. Transforming growth factor beta (TGF*β*) controls numerous functions of the human body, including cell proliferation, differentiation, and migration. Thus, this study is aimed at evaluating whether genetic polymorphisms in *TGFB1* and its receptor *TGFBR2* are associated with mandibular retrognathism in German children and adolescents. Children and teenagers older than 8 years in the mixed or permanent dentition were included in this study. Patients with syndromes and facial trauma and patients with congenital alterations were excluded. Digital cephalometric tracings were performed using the anatomical landmarks point A, point B, sella (S), and nasion (N). Patients that have a retrognathic mandible (SNB < 78°) were selected as case group, and the patients with an orthognathic mandible (SNB = 78°– 82°) were selected as the control group. Genomic deoxyribonucleic acid (DNA) from saliva was used to evaluate four genetic polymorphisms in *TGFB1* (rs1800469 and rs4803455) and *TGBR2* (rs3087465 and rs764522) using real-time PCR. Chi-square or Fisher exact tests were used to compare gender, genotype, and allele distribution among groups. Genotype distribution was calculated in an additive and recessive model. Haplotype analysis was also performed. The established alpha of this study was 5%. A total of 146 patients (age ranging from 8 to 18 years) were included in this epidemiological genetic study. The genetic polymorphism rs3087465 in *TGFBR2* was associated with mandibular retrognathism. Carrying the AA genotype in the rs3087465 polymorphism decreased the chance of having mandibular retrognathism (odds ratio = 0.25, confidence interval 95% = 0.06 to 0.94, *p* = 0.045). None of the haplotypes was associated with mandibular retrognathism (*p* > 0.05). In conclusion, we found that the genetic polymorphism rs3087465 in the promoter region of the *TGFBR2* was associated with mandibular retrognathism in Germans.

## 1. Introduction

There are a wide variety of skeletal malocclusions (dentofacial deformities) in humans [1], and the frequency of each dentofacial deformity ranges according to the studied population/ethnicity [2]. One of the most common dental facial deformities is mandibular retrognathism [3], which is a facial alteration of the skeletal jaw-cranial base relationship. Retrognathism is characterized by a retruded position of the mandible as a result of an anomaly of the skeletal jaw-cranial base relationship [4]. This condition has a strong genetic background and some genes have been associated with mandibular retrognathism in humans from different populations in past years [3–6]. Some previous studies associated mandibular retrognathism with genetic polymorphisms in genes encoding *Myosin IH* (*MYO1H*) [5], *Matrilin 1* (*MATN1*) [4], *bone morphogenetic protein 2* (*BMP2*) [7], *ADAM metallopeptidase with thrombospondin type 1 motif 9* (*ADAMTS9*) [6], and *parathyroid hormone* (*PTH*) and the vitamin-D-related genes: *vitamin D receptor* (*VDR*), *cytochrome P450 family 24 subfamily A member 1* (*CYP24A1*), and *cytochrome P450 family 27 subfamily B member 1* (*CYP27B1*) [8].

The transforming growth factor beta (TGF*β*) family constitutes a group of three isoforms, TGF*β*1, TGF*β*2, and TGF*β*3. Their structure is formed by interrelated dimeric polypeptide chains. Pleiotropic and redundant functions of the TGF*β* family control several functions, such as cell proliferation, differentiation, and migration in all human tissues. The TGF*β* family has numerous key roles in the bone tissue controlling physiological phenomena regarding maintenance of metabolic homeostasis [9]. TGF*β* isoforms and their receptors, type I receptor (TGF*β*RI or ALK5) and type II receptor (TGF*β*RII or TGFBR2) play innumerous essential roles in endochondral and intramembranous ossification [10].

Several functional genetic polymorphisms were identified in TGFB1 (gene encoding TGF*β*1) and TGFBR2 (gene encoding TGF*β*RII) and they were associated with higher serum or plasma level of TGF*β*1 and enhanced transcriptional activity of TGF*β*RII [11]. It is possible that some of these functional genetic polymorphisms play a role in the establishment of maxillary and mandibular morphology leading to skeletal malocclusion phenotypes. Therefore, the present study evaluated if well-known functional genetic polymorphisms in *TGFB1* and its receptor *TGFBR2* are associated with mandibular retrognathism in Germans children and teenagers.

## 2. Materials and Methods

This study was approved by the Ethics Committee from the University of Regensburg (# 19-1549-101). Informed consent was obtained from all patients and/or their legal guardians (in the case of minors during the sample collection), and age-appropriate assent documents were also used for patients younger than 14 years. This project was made following the Helsinki Declaration. The Strengthening the Reporting of Genetic Association study (STREGA) statement checklist was followed to design the study and report the results. The chi-square test for sample size (power) calculation was performed by PASS 15 Power Analysis and Sample Size Software (NCSS, LLC. Kaysville, Utah, USA). Küchler et al.'s (2021) study was used to obtain the *W* effect size (0.225), with an alpha of 5% and power of 80% the test predicts 155 patients for this study.

This is a cross-sectional nested case-control study design. For this cross-sectional study, patients undergoing orthodontic treatment at private orthodontic practices in Regensburg-Germany and the University of Regensburg were screened. Children and teenagers of both sexes were recruited and they were consecutively included in this study from 2020 to 2021.

Patients with underling syndromes, adults (older than 18 years), patients with mandibular prognathism and congenital alterations including tooth agenesis (except for third molar agenesis), oral cleft patients, and patients with facial trauma were excluded. Only one patient per family was recruited. To minimize genetic and phenotypic variance and to maximize data interpretability, only patients with a Middle-European ancestry (at maximum one grandparent not from Middle Europe) were included. All patients included were children older than 8 years in the mixed or permanent dentition.

### 2.1. Retrognathic and Orthognathic Characterization

Digital lateral cephalograms from each patient's orthodontic record with the mandible in centric relationship were evaluated in this study.

The measurements were performed by two trained and calibrated examiners. Intraclass correlation coefficients (ICC) were used to calculate intra- and interexaminer reliability. Interexaminer reliability showed significant good agreement for both examiners (ICC, 0.98 - 0.95). Intraexaminer reliability also showed significant good agreement (ICC, 0.97 - 0.91).

Digital cephalometric were tracings performed using the software Ivoris® (Computer konkret AG, Falkenstein, Germany, version 8.2.15.110). The anatomical landmarks point A, point B, sella (S), and nasion (N) were determined manually using the cephalometric analysis software, and, subsequently, the angular measurements SNB and ANB were calculated (Figure 1).

Patients presenting a retrognathic mandible (SNB < 78°) were selected as a case group, while those presenting an orthognathic mandible (SNB = 78°– 82°) were selected as a control group. Patients having mandibular prognathism (SNB > 82°) were excluded.

### 2.2. Selection of Genetic Polymorphisms and Laboratorial Analysis

For the selection of the genetic polymorphisms, we searched the promoter, intronic, and coding genetic polymorphisms of the *TGFB1* and *TGFBR2* from the dbSNP database (http://www.ncbi.nlm.nih.gov/snp/). Only genetic polymorphisms with heterozygosity above 0.2 in the global population were considered. The classification of each genetic polymorphism as potentially functional (polymorphisms that can result in amino acid changes of the corresponding proteins or occurring in the promoter region of the gene and potentially affecting the expression of the gene or previously associated with other conditions and potentially clinically relevant) was also taken into consideration in the selection process. The characteristics and description of the genetic polymorphisms selected for this study are presented in Table 1.

For the genotyping analysis, we used genomic DNA that was isolated from buccal epithelial cells collected using two cytobrushes placed in extraction solution (Tris-HCl 10 mmol/L, pH 7.8; EDTA 5 mmol/L; SDS 0.5%, 1 mL). Briefly, proteinase K (100 ng/mL) were added to each tube. Ammonium acetate was added to eliminate nondigested proteins, and the liquid was then centrifuged. DNA was precipitated with isopropanol, washed with ethanol. The DNA was quantified by spectrophotometry (Nanodrop 1000; Thermo Scientific, Wilmington, DE, USA) [12].

The selected genetic polymorphisms, which were described in Table 1, were blindly genotyped via real-time polymerase chain reaction (PCR) using the Mastercycler® ep realplex-S thermocycler (Eppendorf AG, Hamburg, Germany). The TaqMan technology was used. Initial denaturation at 95°C for 30 seconds, followed by 40 cycles of denaturation at 92°C for 5 seconds and annealing/extension at 60°C for 20 seconds. The 3.125 *μ*L reaction volume contained 1.5 *μ*L Master Mix, 0.125 *μ*M TaqMan probe, and 4 ng DNA in 1.5 *μ*M nuclease-free water. Assays and reagents were supplied by Applied Biosystems (Foster City, CA, USA). A negative control template was included in each reaction (each 96-well plate), in which the reaction mixture contains the reagents, but not the DNA. Additionally, 10% of the samples were randomly selected in order to repeat the analysis and showed 99% concordance.

Patients with not enough DNA or DNA samples that failed to be genotyped in the PCR analysis were excluded from the further analyses.

### 2.3. Statistical Analysis

Chi-squared test estimated the Hardy-Weinberg equilibrium (HWE) for each studied polymorphism (https://wpcalc.com/en/equilibrium-hardy-weinberg/).

Chi-squared or Fisher's exact tests compared gender, genotype, and allele distribution among groups and genotype distribution was calculated in an additive model and recessive model. Haplotype analysis was also performed. PLINK version 1.06 (https://zzz.bwh.harvard.edu/plink/ld.shtml) was used for the analysis with an established alpha of 5% (*p* < 0.05). The odds ratio and confidence interval 95% was calculated to investigate the chance of presenting mandibular retrognathism for the associated genetic polymorphism.

## 3. Results

A total of 168 patients were screened, two patients were excluded due to biological relations to included patients (siblings), one due to oral cleft, 13 due to age older than 18 years, and six patients due to mandibular prognathism. Finally, 146 patients (age ranging from 8 to 18 years) were included in this epidemiological genetic study. The characteristics of the included sample are presented in Table 2. Mean age in the mandibular retrognathism group was 11.56 years (standard deviation = 2.05), while the mean age in the mandibular retrognathism group was 12.66 years (standard deviation = 2.2). The SNB angle was significantly lower in the mandibular retrognathism group (ranging from 66.0° to 77.9°) than in the control group (ranging from 78.1° to 81.9°) (*p* = 0.0014).

All the genetic polymorphisms assessed were within the Hardy-Weinberg equilibrium (chi‐square^HWE^ = 0.452 for rs1800469, chi‐square^HWE^ = 0.309 for rs4803455, chi‐square^HWE^ = 3.17 for rs3087465, and chi‐square^HWE^ = 0.161 for rs764522). For the rs1800469 (A/G), rs4803455 (C/A), rs3087465 (A/G), and rs764522 (G/C) polymorphisms, success rates of genotyping were 95.9%, 90.4%, 95.9%, and 91.8%, respectively.

Table 3 shows the genotype and allele distributions and the association results in the allele distribution and genotype distribution in additive and recessive models. The only significantly associated polymorphism was rs3087465 in *TGFBR2*. Patients that carry the AA genotype in the polymorphism rs3087465 had significantly decreased the chance to have mandibular retrognathism (odds ratio = 0.25, confidence interval = 0.06 to 0.94, *p* = 0.045).

The haplotype analysis for the polymorphisms in *TGFB1* (rs4803455-rs1800469) and *TGFBR2* (rs764522-rs3087465) is presented in Table 4. There was no statistically significant association (*p* > 0.05).

## 4. Discussion

Some studies evaluating dentofacial deformities via cephalometric images in different populations/ethnicities have been performed in the past decades to investigate the genetic contribution of different skeletal malocclusions. Literature reviews showed that many genes involved in a range of functions are associated with skeletal malocclusions [13, 14], especially genes encoding growth factors and growth factor receptors [8, 15–17]. Growth factors are found in all tissues; they regulate local cell-to-cell metabolism and mediate cellular effects of different hormones. Bone matrix is a large reservoir for numerous growth factors that are regulators of bone remodeling processes [18]. Therefore, we hypothesized that functional genetic polymorphisms in *TGFB1* and *TGFBR2* could be involved in the etiology of mandibular retrognathism in Germans.

In our study, we explored two well-known genetic polymorphisms in *TGFB1*. Several polymorphisms have been described in the coding and regulatory sequences of the *TGFB1* gene, including a promoter polymorphism involving a cytosine-to-thymine transition. The -509C/T functional promoter polymorphism (rs1800469) within the *TGFB1* gene has been extensively assessed in different genetic epidemiological studies. Moreover, a number of studies have attempted to investigate whether the polymorphic variants in *TGFB1* change TGF*β*1 expression [19–21]. Another genetic polymorphism widely explored in different conditions is rs4803455 involving a C-to-A transition, which is located in intron 2 of *TGFB1* and was therefore selected in our study. Although both variants (rs1800469 and rs4803455) with a known role were hypothesized as potential candidates for mandibular retrognathism, none of these genetic polymorphisms were associated with the phenotype in our study. However, it is possible that other polymorphisms in these genes could be involved in mandibular retrognathism.

TGFB initially binds its receptor, which is TGFBR2 and later transactivates TGFBR1, leading to the formation of a heterotetrameric receptor complex. TGFBR1 and TGFBR2 are members of the serine-threonine protein kinase family. TGFBR2 is a constitutive kinase, while TGFBR1 kinase is only activated after the formation of the TGFB/TGFBR2 complex [22]. Recently, there have been several studies investigating the association between genetic polymorphisms in *TGFBR2* in various diseases, such as abdominal aortic aneurysm, papillary thyroid carcinoma, and end-stage renal disease, especially two promoter polymorphisms rs764522 (-1444C/G) and rs3087465 (-834A/G) [23–25]. Therefore, we decided to investigate these polymorphisms in our study. We observed that the AA genotype in polymorphism rs3087465 (-834A/G) acted as a protective factor for mandibular retrognathism. Interestingly, this genetic polymorphism located in a promoter region was previously associated with alterations in TGF*β* type II receptor expression [26–28].

Although the sample size was a limitation that could lead to a type I error, our results raised a possibility of a novel candidate gene for mandibular retrognathism. It is interesting to mention that mutations in the *TGFBR2* gene are associated with Marfan syndrome [29] and Loeys-Deitz syndrome [30]. The craniofacial phenotypes of these both syndromes included mandibular retrognathism as a common trait observed [31–33], which clearly suggests the role of genetic polymorphisms in *TGFBR2* in nonsyndromic mandibular retrognathism. Also, studies with animal models have demonstrated that TGFBR2 plays a critical role in the formation of the intramembranous bone and endochondral bone and that TGFBR2 is crucial for skeletal development [34, 35] including craniofacial development [34, 36, 37]. Deletion of *Tgfbr2* via Col2a1-Cre in mice caused several defects in the base of the skull [34]. Removal of TGFBR2 driven by Prx-Cre results in defects in the skull vault [37]. Mice with *Tgfbr2* conditional gene ablation in the cranial neural crest have craniofacial anomalies including defects in mandibular development resulting in a smaller mandible [36].

To the best of our knowledge, this is the first study to investigate genes involved in mandibular retrognathism in Germans; however, it is important to emphasize that these findings must be validated in independent larger cohorts. Another important aspect to be discussed is that we investigated children and teenagers. This approach was also performed before. The study from Sasaki et al. [15] investigated the association between a genetic polymorphism in the gene encoding growth hormone receptor (GHR) and mandibular prognathism in children aged 3 to 13 years. The authors concluded that P561T in GHR may affect mandibular growth during early childhood.

Briefly, our results add novel information regarding the genetic contribution to mandibular retrognathism etiology suggesting rs3087465 (-834A/G) in TGFBR2 as candidate gene, additionally to the previously genes suggested in studies from different populations: *MYO1H* [5], *MATN1* [4], *BMP2* [7], *ADAMTS9* [6], *PTH*, *VDR*, *CYP24A1*, and *CYP27B1* [8]. Once our understanding of the nature of the genetic influences improves, we will be able to provide a clearer idea of how genes and environmental factors interact to influence mandibular retrognathism in humans.

## 5. Conclusion

The genetic polymorphism rs3087465 in the promoter region of the *TGFBR2* was associated with mandibular retrognathism in Germans. Determining the factors affecting mandibular growth will contribute to early diagnosis and treatment of mandibular retrognathism.

## Figures and Tables

**Figure 1:** Lateral cephalometric landmarks and reference lines studied. Points: point A, point B, sella (S), and nasion (N).

**Table 1:** Characteristics of the studied genetic polymorphisms.

Gene	Polymorphism and base change	Comments
*TGFB1* *Transforming growth factor beta 1*	rs1800469 (T/C)	Polymorphism rs1800469 is located in the promoter region of the TGFB1 gene and has the function of regulating expression levels of protein TGF*β*1 (affects gene transcriptional activity and serum levels of TGF*β*1) [19, 20].
	rs4803455 (C/A)	The polymorphism rs4803455 is located in intron 2 of TGFB1 gene and was associated with a variety of different conditions (https://www.ncbi.nlm.nih.gov/snp/rs4803455). Moreover, it was suggested as a potential genetic marker for growth response to recombinant human growth hormone (r-hGH) treatment [38].

*TGFBR2* *Transforming growth factor beta receptor 2*	rs3087465(A/G)	Polymorphism rs3087465 is located in the promoter region of the gene and increases TGF*β* type II receptor expression [26].
	rs764522 (G/C)	The polymorphism rs764522, which is located in 5 kb upstream in the promoter region of *TGFBR2* increases TGF*β* type II receptor expression [26].

**Table 2:** Comparison of cephalometric variables between mandibular retrognathism and orthognathic mandible.

Variables	Orthognathic mandible (*n* = 50)	Mandibular retrognathism (*n* = 96)	*p* value
*Gender,n(%)*			
Male	29 (58.0%)	45 (46.8%)	0.202
Female	21 (42.0%)	51 (53.2%)	
*SNB (°)*			
Mean (SD)	79.62 (SD 1.07)	78.32 (SD 2.67)	0.001∗
*ANB (°)*			
Mean (SD)	3.48 (SD 2.75)	4.26 (SD 2.27)	0.068

Note: SD: standard deviation; ^∗^statistically significant difference (*p* < 0.05); *n*: number of individuals; %: percent; °: degrees.

**Table 3:** Genotype distribution among group and *p* values.

Gene	rs	Genotype distribution and allele distributions, *n* (%)			*p* value^Genotype^	*p* value^Allele^	*p* value^Recessive^
		Genotype	Orthognathic mandible	Mandibular retrognathism			
*TGFB1*	rs1800469	TT	5 (10.0)	4 (4.4)	0.310	0.525	0.199
		CT	18 (36.0)	41 (45.6)			
		CC	27 (54.0)	45 (50.0)			
		A	28 (28.0)	49 (27.2)			
		G	72 (72.0)	131 (72.8)			
	rs4803455	CC	10 (20.8)	18 (21.4)	0.740	0.692	0.478
		CA	27 (56.3)	42 (50.0)			
		AA	11 (22.9)	24 (28.6)			
		C	47 (48.0)	78 (46.4)			
		A	49 (52.0)	90 (57.3)			

*TGFBR2*	rs3087465	AA	6 (12.0)	3 (3.3)	0.098	0.603	0.045∗
		AG	21 (42.0)	48 (53.3)			
		GG	23 (46.0)	39 (43.3)			
		A	33 (33.0)	54 (30.0)			
		G	67 (67.0)	126 (70.0)			
	rs764522	GG	0 (0.0)	2 (2.3)	0.575	0.525	0.302
		GC	11 (23.9)	22 (25.0)			
		CC	35 (76.1)	64 (72.7)			
		G	11 (12.0)	26 (14.8)			
		C	81 (88.0)	150 (85.2)			

Note: ^∗^means statistically significant difference; *n*: number of individuals; %: percent; rs: the code of polymorphisms; *TGFB1*: transforming growth factor beta 1; *TGFBR2*: transforming growth factor beta receptor 2; C: cytosine; A: adenine; T: thymine; G: guanine.

**Table 4:** Haplotype analysis of the studied genetic polymorphisms.

Gene	Haplotype		Frequency		*p* value
			Orthognathic mandible	Mandibular retrognathism	
*TGFB1*	rs4803455-rs1800469	CT	0.264	0.242	0.706
		AT	0.027	0.025	0.930
		CC	0.225	0.213	0.818
		AC	0.482	0.517	0.586

*TGFBR2*	rs764522-rs3087465	GA	0.084	0.103	0.610
		CA	0.252	0.208	0.407
		GG	0.035	0.049	0.602
		CG	0.627	0.639	0.855

Note: *TGFB1*: transforming growth factor beta 1; *TGFBR2*: transforming growth factor beta receptor 2; C: cytosine; A: adenine; T: thymine; G: guanine.

## Data Availability

The data generated during the current study are available from the corresponding author on reasonable request.
